The article "In Vitro and In Vivo Analysis of the Effects of 3D-Printed Porous Titanium Alloy Scaffold Structure on Osteogenic Activity" was published in 2022. Journal: Biomed Res Int.

# In Vitro and In Vivo Analysis of the Effects of 3D-Printed Porous Titanium Alloy Scaffold Structure on Osteogenic Activity

**DOI:** 10.1155/2022/8494431

**Published:** 2022-08-13

**Authors:** Zhenchao Xu, Yilu Zhang, Yunqi Wu, Zhen Zhang, Dingyu Jiang, Runze Jia, Xiyang Wang, Zheng Liu

**Affiliations:** ^1^Department of Spine Surgery and Orthopaedics, Xiangya Hospital of Central South University, 87# Xiangya Road, Changsha, Hunan 410008, China; ^2^Hunan Engineering Laboratory of Advanced Artificial Osteo-Materials, 87# Xiangya Road, Changsha, Hunan 410008, China; ^3^Department of Orthopedics, Hunan Children's Hospital, 86# Ziyuan Road, Changsha, Hunan 410007, China

## Abstract

The effect of titanium scaffold geometry on the bone regeneration ability of the scaffold remains unclear. Here, selective laser melting as a 3D printing technology was used to create porous titanium alloy scaffolds with two unit structures: a hollow hexagonal prism (group A) and a hollow triangular prism (group B). The structures and morphologies of the scaffolds were characterized before mechanical properties were simulated. Cell adhesion behaviors, osteoblast activity and proliferation, and alkaline phosphatase (ALP) activity were evaluated, in addition to in vivo testing in an animal model. The results showed that the two scaffolds made of Ti6Al4V had compression moduli similar to that of human cortical bone (116.91 ± 0.01 and 174.29 ± 2.21 MPa vs. 89–164 MPa). The two scaffolds were nontoxic to cells and had good biocompatibility, while group A scaffolds facilitated cell adhesion. The number of cells increased gradually in culture. The ALP activity of cells on group A scaffolds demonstrated higher osteogenic ability than that of group B scaffolds. The in vivo tests showed that all scaffolds retained their shape well after implantation, and no obvious inflammatory reaction or infection in surrounding tissues was found. Based on fluorescence staining, mature new bone formation was found at week 12. Group A scaffolds showed better bone integration ability compared with group B scaffolds. The percentage of new bone area in group A (7.5%) was higher than that in group B (6.5%). This research suggests that the hollow hexagonal prism structure of porous scaffolds can promote osteogenic differentiation and osseointegration better than the triangular prism structure.

## 1. Introduction

Bone repair scaffolds must have at least the following characteristics [1–3]: (1) good biocompatibility, (2) mechanical properties suitable for host tissue, and (3) a highly porous and interconnected structure that allows cell migration, proliferation, differentiation, and exchange of nutritional waste. Therefore, it is necessary to study the effects of the morphological parameters of these scaffolds, such as the influence of pore shape, pore size, and permeability on biocompatibility.

The article "In Vitro and In Vivo Analysis of the Effects of 3D-Printed Porous Titanium Alloy Scaffold Structure on Osteogenic Activity" was published in 2022. Journal: Biomed Res Int.

Scaffolds should have evenly distributed and connected large pores as well as high porosity. On one hand, this ensures infiltration of cells, diffusion of nutrients, and removal of waste. On the other hand, it provides space for the formation of vascular tissue and new bone. Compared with other scaffolds with larger pore sizes, scaffolds with pore sizes between 300 *μ*m and 400 *μ*m have shown better performance [4]. In another report [5], 200–500 *μ*m is considered to be ideal pore size to promote bone regeneration and blood vessel formation.

Titanium and its alloys offer good biocompatibility, excellent corrosion resistance, and low tissue reactivity. Titanium alloy also has the advantages of a nondegradable and stable structure that is preserved over the long term, which is suitable for hard tissue replacement. The good biocompatibility of titanium implants may be related to the natural formation of thin titanium dioxide sheets with a thickness of 1.8–17 nm on the titanium surface [6]. Natural titanium dioxide is considered an inert biomaterial because of its difficulty in forming direct chemical bonds with bone tissue. Therefore, various surface modification methods have been used to improve the biological activity of titanium and its alloys. Some studies have found that acid or base treatment improves the biological activity and bone regeneration of titanium [7–12].

Additive manufacturing (AM), also known as 3D printing technology, has become an innovative material processing method that is used to promote the manufacture of bone tissue engineering scaffolds, which have afforded revolutionary development of traditional treatment methods for large bone defects [13]. Using existing materials, 3D printing technology seeks to develop innovative scaffolds that provide satisfactory mechanical properties for the repair of load-bearing bones [14]. In addition, based on medical image data, 3D printing technology can directly manufacture patient-specific bone substitutes with complex structures from biomaterials and enable the precise design of structures at both macro- and microscales to provide optimal in vivo responses, such as enhancement of bone regeneration by bone conduction [15]. Selective laser melting (SLM) is a 3D printing technology. Under high-energy laser, metal powder is completely melted, cooled, and solidified and then metallurgically welded with base metal, before accumulation layer by layer to form a three-dimensional solid. In terms of medical treatment, SLM can directly manufacture metal scaffolds to promote bone regeneration for load-bearing [16]. Among all metal materials, titanium and its alloys have good biocompatibility, high wear resistance, strength-weight ratio, low elastic modulus, and excellent corrosion resistance, which enable them to be used as scaffolds for bone growth and reconstruction for weight-bearing bone defects [17].

The article "In Vitro and In Vivo Analysis of the Effects of 3D-Printed Porous Titanium Alloy Scaffold Structure on Osteogenic Activity" was published in 2022. Journal: Biomed Res Int.

To date, a variety of 3D porous titanium scaffolds have been developed in many preclinical and clinical studies through 3D printing technology, and their properties have been significantly improved [6]. The size and geometry of pores as well as porosity are important properties of porous titanium scaffolds for bone regeneration. In a previous study, pore scaffolds having six different geometries were created, and pore shape was shown to affect the permeability, stiffness, strength, and stress concentration of Ti6Al4V bone scaffolds [18]. Square pores were found to facilitate cell growth [19]. In addition, a pore size of 650 *μ*m was more beneficial for bone growth than the sizes of 400–500 *μ*m and 1100 *μ*m [20]. Such optimal size was also found in another study in which porous scaffolds with a pore diameter of 700–200 *μ*m showed better bone regeneration capacity than those with pore diameters of 500 and 1500 *μ*m [21, 22].

In this study, two groups of porous titanium alloy scaffolds were prepared with Ti6Al4V powder by 3D printing SLM technology to further explore the effect of scaffold structures. The 3D-printed titanium alloy porous scaffolds had different unit structures, one of which was a hollow hexagonal prism (group A) and the other was a hollow triangular prism (group B). After morphology characterization and mechanical property simulation, in vitro and in vivo experiments were performed to evaluate the osteogenic abilities of the two scaffolds.

## 2. Materials and Methods

Two scaffolds with different geometries (hollow hexagonal prism and hollow triangular prism) were created using SLM technology. The structures and morphologies of the scaffolds were characterized before mechanical properties were stimulated. In vitro experiments were performed, including cell adhesion, morphology observation, osteoblast activity and proliferation evaluation, and ALP activity test. Rabbits were used in in vivo experiments. X-ray and microcomputed tomography (CT) examinations were performed, while bone tissue formation was characterized by fluorescence staining.

A flow chart of the study is shown in Scheme 1.

### 2.1. Selective Laser Melting (SLM) Technology

With the help of SOLIDWORKS CAD software (Dassault Systèmes, France), 3D data models of porous titanium alloy scaffolds with two kinds of unit structures were designed (Figures 1(a) and 1(b)). Metal laser melting equipment (Hunan Farsoon High-Technology Co., Ltd.) was used to create the designed scaffolds of Ti6Al4V (TC4) powder (Research Institute of Powder Metallurgy, Central South University, China). The porous scaffolds were taken out from the 3D printing device, and the unmelted metal powder in the scaffold was blown away with an air gun. Ultrasonic cleaning was performed for 10 min successively with acetone, anhydrous ethanol, and deionized water (residual toxic metal particles were cleaned). The porous titanium alloy scaffolds were placed in 5 mol/L NaOH solution at 60°C for 24 h and then repeatedly cleaned with deionized water before drying. The porous scaffolds were then placed in 0.5 mmol/L HCl solution at 70°C for 24 h and then repeatedly cleaned with deionized water before drying. The scaffolds were finally put into a sintering furnace (FCT Systems, Germany) and heated to 600°C at 5°C/min, before atmospheric annealing for 1 h.

The article "In Vitro and In Vivo Analysis of the Effects of 3D-Printed Porous Titanium Alloy Scaffold Structure on Osteogenic Activity" was published in 2022. Journal: Biomed Res Int.

### 2.2. Simulation

The 3D data model of the 3D-printed porous titanium alloy support was imported into the ANSYS software to complete the creation of the finite element geometric model, set the material properties used in the calculation model, and apply the acting load on the finite element to simulate the stress of the support. The porous scaffold was placed in the biomechanical tester for biomechanical testing of the scaffold. We also added Figure 1(c) to show how the finite element analysis software ANSYS simulates the stress of the support.

### 2.3. Characterizations

#### 2.3.1. Structures and Morphologies

The scaffold samples were cleaned with anhydrous ethanol and deionized water using an ultrasonic machine (Shanghai Yijing Ultrasonic Instrument Co., Ltd.) for 10 min successively. The microstructures of the titanium scaffolds were detected by scanning electron microscopy (SEM) (Czech FEI Company), and the surface elements were analyzed by energy spectrum analysis (EDS) and X-ray diffraction (XRD) (Bruke Germany Company).

#### 2.3.2. Preparation of Cell Suspension

MC3T3-E1 osteogenic precursor cell suspension (Cell Resource Center, Shanghai Institutes of Biological Sciences, Chinese Academy of Sciences, China) was cultured in *α*-Minimal Essential Medium (*α*-MEM, HyClone, USA) containing 10% fetal bovine serum (Gibco, USA) and 1% double antibody (streptomycin and penicillin were both 100 U/mL, HyClone, USA) in a 5% CO_2_ cell incubator at 37°C, and the medium was changed every 2 days. The cells were digested and subcultured. The number of cells was measured by a cell counting apparatus (Wuhan Bailezhen Biotechnology Co., Ltd.), and then, the required concentration of cell suspension was prepared by adding culture medium.

The article "In Vitro and In Vivo Analysis of the Effects of 3D-Printed Porous Titanium Alloy Scaffold Structure on Osteogenic Activity" was published in 2022. Journal: Biomed Res Int.

#### 2.3.3. Observation of Cell Adhesion

The scaffolds of groups A and B were disinfected and placed in 48-well plates with 3 samples in each group. A small amount of complete medium was added and soaked overnight. The medium was sucked out the next day, and cells were inoculated. The number of cells was measured with a cell counter, and then, the medium was added to prepare the cell suspension with a concentration of 2 × 10^6^ cells/mL. Next, 100 *μ*L per well cell suspension was added over the surface of the material, and 700 *μ*L was added to cover the surface of the material.

The culture plate was placed in a 5% CO_2_ incubator at 37°C. After the cells and the scaffold were cultured for 24 h, the culture plate was removed, the medium was sucked and discarded, and the scaffolds were gently blown and washed with phosphate-buffered saline (PBS) 3 times. The scaffolds were gently moved into a new 24-well plate with microscopic tweezers, and 1 mL of 4% paraformaldehyde solution (New Cell & Molecular Biotech Co., Ltd., USA) was added to each well for fixation for 5 min. After rinsing with PBS, 50 *μ*g/mL DAPI solution (Sigma) was added to the surface of the scaffold to stain the nuclei for 5 min. After staining, PBS solution was added to shake the nuclei for 3 times, each time for 10 min. The whole staining process was shielded from light. After staining, the Petri dish was placed under a fluorescence microscope (Nikon, Japan). Five fields were randomly selected, and the cell count was quantified.

#### 2.3.4. SEM Observation

After inoculation, the 48-well culture plates were placed in a 37°C, 5% CO_2_ incubator, and the liquid was changed every 2 days. After 48 h of culture, the medium was discarded, and PBS solution was added to the material for three times. After the PBS was discarded, 2.5% glutaraldehyde (Leagene Biotechnology) precooled at 4°C was added and fixed for 4 h (stored in a refrigerator at 4°C). Glutaraldehyde was absorbed, dehydrated by 50% ~100% (twice) gradient ethanol (15 min/time), and dried. The cell surface morphology was observed using SEM.

#### 2.3.5. Osteoblast Activity

The effects of 3D-printed titanium alloy porous scaffolds (3 samples per group) on osteoblast activity were detected using a live and dead cell viability/toxicity detection kit (KeyGen Biotech). After 3 days of culture, the cells were stained for viability/toxicity.

#### 2.3.6. Osteoblast Proliferation

At 1, 3, 5, and 7 days, the CCK-8 reagent (DOJINDO, Japan) was mixed and diluted with the culture medium at a ratio of 1 : 10. The culture medium in each well was discarded, and 800 *μ*L of diluted CCK-8 reagent was added in each well that was put into the incubator for further cultivation of 4 h. The supernatant from each well was carefully collected and transferred to a 96-well plate. Then, the absorbance (optical density (OD)) at 450 nm was measured with a microplate (BioTek, USA) and recorded.

The article "In Vitro and In Vivo Analysis of the Effects of 3D-Printed Porous Titanium Alloy Scaffold Structure on Osteogenic Activity" was published in 2022. Journal: Biomed Res Int.

#### 2.3.7. ALP Activity

After 1 day of culture, the medium was changed to osteogenic induction medium (*α*-MEM + *β*-sodium glycerophosphate+ascorbic acid), which was placed into a cell culture box (Cymerfeld, USA) for culture, and the medium was changed every 3 days. On the 12th day of culture, the medium was discarded and gently rinsed with PBS 3 times. 200 *μ*L 1% Triton X-100 (Shanghai Solarbio Bioscience & Technology Co., Ltd., China) PBS buffer was added into each well to lysis cells. Then, the supernatant was centrifuged, and ALP activity was quantitatively detected by an ALP detection kit (Beyotime Biotechnology).

#### 2.3.8. Rabbit Femur Defect Repair In Vivo

Ethical approval from the Ethics Committee of Xiangya Hospital affiliated to Central South University was obtained for the animal study (No. 201603243). Male New Zealand rabbits (Hunan Taiping Biological Technology Co., Ltd.) were selected as experimental animals. The animals were of ordinary grade, weighing about 3 kg, and aged 5 months. They were purchased from the Department of Experimental Animal Science, Central South University. All animals were fed in strict accordance with the standards. Twelve male New Zealand rabbits were randomly divided into 2 groups with 6 rabbits in each group.

New Zealand rabbits were weighed and anesthetized with 3% sodium pentobarbital (1 ml/kg) by ear vein injection. After successful anesthesia, the hair around the left femoral condyle was removed with an animal hair shaver. The rabbit was placed in the right decubial position flat on the operating table for fixation and then disinfected. Sterile towels were spread, and a longitudinal incision was made at the distal end of the left femur. After the skin was cut, the fascia and muscle were separated layer by layer, and the periosteum was stripped until the lateral condyle of the femur was completely exposed. The area about 4 mm away from the articular surface was marked, and the medical electric drill was installed. The cylindrical bone defect area with a diameter of 5 mm and a depth of 10 mm was prepared by successively expanding the hole with a diameter of 2 mm with a Kirschner needle and 3 mm, 4 mm, and 5 mm drill bits. During the drilling process, normal saline was used to wash and cool down. After drilling, hydrogen peroxide and normal saline were used to wash the bone defect area successively, and the bone debris in the area was cleaned. Then, the scaffold in each group was implanted into the defect area. The incision was sutured layer by layer and disinfected with iodine. Cefoxitin was injected for 3 consecutive days after surgery. The general condition and wound healing of the animals were observed regularly after operation.

The article "In Vitro and In Vivo Analysis of the Effects of 3D-Printed Porous Titanium Alloy Scaffold Structure on Osteogenic Activity" was published in 2022. Journal: Biomed Res Int.

The animals to be killed were injected with calchloflavin solution 14 and 4 days before postoperative sampling. For this, 400 mg calceoflavin was dissolved in 50 mL normal saline. First, 1 g sodium bicarbonate was added to make the calceoflavin completely dissolve, and the solution was filtered for sterilization. The left femoral condyle was removed, and the soft tissue on the surface of the specimen was removed. The specimen was fixed with 80% alcohol and stored at 4°C under dark conditions.

#### 2.3.9. X-Ray and Micro-CT Examination

The specimens in each group were examined by plain X-ray film, followed by micro-CT scanning with a voltage of 70 kV and a current of 141 *μ*A. The scanning range was 360°, and the thickness of tomography was 18 *μ*m. Ctan software was used for 3D reconstruction, and the region within the underside of the scaffold was selected as the region of interest by software scanning, and the data of new bone tissue in the pores of the porous scaffold were obtained through gray analysis, including (1) trabecular thickness (Tb.Th), (2) trabecular number (Tb.N), and (3) bone volume fraction (BV/TV) = bone trabecular volume (BV)/total volume (TV).

After micro-CT examination, all samples were immersed in 10% formalin solution for 24 h, 70% alcohol for 2 h, 95% alcohol for 20 h, and 100% alcohol for 2 h and then dried for 6 h. After treatments to solidify protein and prevent corrosion, followed by dehydration and drying, the samples were immersed in a glass tube containing polymethyl methacrylate monomer, immersed in a low vacuum for 30 min (at this time, no gas emerged), and solidified in a water bath at 27°C. The samples were cut into 200 *μ*m samples with a hard tissue slicer (AKT Company, Germany) and then glued to the resin sheet with quick-drying adhesive. The sample slices on the resin sheet were ground to 50 *μ*m with a grinding machine and polished. Fluorescence labeling of bone tissue was observed under a laser confocal microscope (CLSM, Zeiss, Germany).

After the staining was completed, the images were observed and collected under an optical microscope. Semiquantitative analysis was performed on the area of new bone tissue in the scaffold using the ImageJ software (NIH, USA). The calculation method was as follows: bone area fraction (%) of each visual field = new bone area/total visual field area × 100%.

The article "In Vitro and In Vivo Analysis of the Effects of 3D-Printed Porous Titanium Alloy Scaffold Structure on Osteogenic Activity" was published in 2022. Journal: Biomed Res Int.

### 2.4. Statistical Analysis

The SPSS24.0 system was used to analyze the experimental data, and the data were expressed as mean ± standard deviation (*X* ± *S*). The independent sample “*t*” test was used to calculate the *P* values for comparative analyses between groups. Data showing any deviation from normal distribution were analyzed using the rank sum test. When *P* < 0.05, the difference was considered statistically significant.

## 3. Results

### 3.1. Preparation and Characterization of 3D-Printed Porous Titanium Alloy Scaffolds

Figure 2 shows the physical images of 3D-printed porous titanium alloy scaffolds prepared by SLM technology. The general shape of the porous scaffolds was cylindrical, and they were designed with two specifications: one was 10 mm in diameter and 5 mm in height, and the other was 5 mm in diameter and 10 mm in height, with an internal porosity of 60% and an aperture of 500 *μ*m. In vivo and in vitro tests were carried out to verify their effects on bone integration.

The finite element analysis software ANSYS was used to simulate the stress of the scaffold. The finite element simulation results show that the compression modulus of the scaffold was 116.91 ± 0.01 MPa, which is close to the compression modulus of human cortical bone (89–164 MPa) and helpful for avoiding the stress shielding effect of implants. The axial force of the scaffold was detected by a biomechanical detector, and the result was 174.29 ± 2.21 MPa, which is similar to the compression modulus of human cortical bone (89–164 MPa).

As shown in Figures 3(a) and 3(b), compared with the designed 3D model, the surface morphology of porous scaffolds prepared by SLM was not regular but in a state of protrusion around the hole. Adhesion of a large number of titanium powder particles was found on the inner wall. There was some error between the actual and model in aperture size. The surface shape of the hollow hexagonal prism unit structure was different from that of the designed square, which was close to a circle (Figure 3(a)). Its aperture size was 441.3 ± 63.4 *μ*m. The surface shape of the hollow triangular prism unit structure was consistent with the designed triangle (Figure 3(b)), and its aperture size was 453.6 ± 38.2 *μ*m.  Figure 3(c) shows a layer of irregular microfold network structure on the surface of a porous scaffold, namely, titanium oxide layer. As shown in Figure 3(d), EDS was used to detect element composition on the surface of the 3D-printed titanium alloy porous scaffold, and the presence of element O indicates the formation of the titanium oxide layer on the surface of the scaffolds. XRD results showed that the diffraction peaks of titanium were all *α*-titanium, and titanium in Ti6Al4V was dominated by *α*-titanium (Figure 3(e)).

The article "In Vitro and In Vivo Analysis of the Effects of 3D-Printed Porous Titanium Alloy Scaffold Structure on Osteogenic Activity" was published in 2022. Journal: Biomed Res Int.

### 3.2. Surface Osteoblast Adhesion Results

Figures 4(a) and 4(b) show the results of DAPI staining. The number of cells adhered to the scaffold in group A was greater than that adhered to group B scaffolds after 24 h in culture.  Figure 4(c) shows the quantitative analysis of cell adhesion number. Five fields were randomly selected. Quantitative statistical analysis of cell count showed that the number of scaffold adhered cells in group A was significantly higher than that in group B (*P* < 0.05).

After the scaffolds were implanted and cultured for 48 h, the surface cells of both groups adhered closely to the titanium oxide layer with good spreading, and many filamentous pseudopodia were extended (Figures 4(d) and 4(e)).

As shown in Figures 4(f) and 4(g), the activity of cells was tested using a live and dead cell staining kit. After staining, the fluorescence microscope showed that there were no obvious dead cells in both groups, indicating that the scaffolds in the two groups were nontoxic to the cells and had good biocompatibility. Cell adhesion in group A was greater than in group B.

### 3.3. Proliferation Results of Osteoblasts Adhered to Scaffolds

CCK-8 results for cell proliferation on the two scaffolds are shown in Figure 4(h). With the increase in culture time, the number of cells adhered to the scaffolds in both groups continued to increase, and there was no significant difference in cell values between group A and group B at each time point (*P* > 0.05).

Quantitative results of ALP activity of cells on scaffolds are shown in Figure 4(i). On the 12th day after culture, the ALP activity on group A was higher than that on group B (*P* < 0.05), suggesting that the osteogenic ability of the scaffold in group A was stronger than that in group B.

### 3.4. In Vivo Rabbit Femur Defect Repair

Rabbit femur samples were obtained at the 4th and 12th weeks after scaffold implantation, and X-ray plane examination was performed after fixation (Figure 5(a)). It can be seen that all implanted scaffolds were in good position without loosening, shedding, or displacement, and there was no obvious inflammatory reaction or infection in the surrounding tissues.

Micro-CT scanning results were reconstructed using the Ctan software. The internal bone growth within the scaffolds is shown in Figure 5(b). The white part is the porous titanium alloy scaffold, and the yellow part is the new bone tissue. It can be seen from the 3D diagram of the bottom surface of the porous scaffolds that a small amount of bone grew around and inside the scaffolds in group A and group B at week 4. By week 12, the bone mass of the scaffolds in the two groups was significantly higher than that in week 4, but there was no significant difference between group A and group B. As can be seen from the results of the three bone tissue parameters (Figure 5(c)), there were no significant statistical differences in bone tissue parameters between group A and group B at weeks 4 and 12 (*P* > 0.05), but the data for group A are all higher than those for group B at week 12.

The article "In Vitro and In Vivo Analysis of the Effects of 3D-Printed Porous Titanium Alloy Scaffold Structure on Osteogenic Activity" was published in 2022. Journal: Biomed Res Int.

All specimens after hard tissue sectioning were placed under CLSM to observe the fluorescence labeling of bone tissue, as shown in Figure 5(d). Calcein marks bone tissue formation in green and titanium alloy in black. At the 4th week, the fluorescence brightness of both groups was weak on the whole, and only a small amount of fluorescence was bright, indicating no obvious mature new bone formation. At the 12th week, the fluorescence brightness of the two groups was significantly enhanced compared with that at the 4th week. The fluorescence distribution of the group A was dense, with mature new bone formed, and the fluorescence was strong at the junction with the material. However, the fluorescence distribution of group B was evenly dispersed, and the new bone was not significantly formed. The fluorescence was weak at the junction with the material, suggesting that the scaffolds in group A had better bone integration ability compared with those in group B.

All hard tissue sections were processed for Van Gieson (VG) staining after observation under CLSM and then observed under an optical microscope, as shown in Figure 5(e). Red is mature new bone tissue, gray brown is bone marrow tissue, and black is titanium alloy material. At week 4, a large number of brown-gray bone marrow tissues grew into the internal pores of the scaffolds in both groups, and a small amount of bone marrow tissue turned red. By contrast, bone marrow tissues in the scaffolds of the group A were more densely distributed. At week 12, mature bone tissue was significantly increased in the internal pores of the scaffolds in the two groups. The bone tissue in the internal pores of the scaffolds in group A was closely combined with the material surface, while there were many gaps between the material surface and the bone tissue in group B.

The percentage of new bone area in the scaffold is shown in Figure 5(f). At week 4, there was no significant statistical difference in the percentage of new bone area in the scaffold between the two groups (*P* > 0.05). At week 12, the percentage of new bone area in the scaffold in group A was higher than that in group B (*P* < 0.05).

The article "In Vitro and In Vivo Analysis of the Effects of 3D-Printed Porous Titanium Alloy Scaffold Structure on Osteogenic Activity" was published in 2022. Journal: Biomed Res Int.

## 4. Discussion

The reason for preparing porous scaffolds instead of solid scaffolds is not only to ensure infiltration of cells, diffusion of nutrients, removal of wastes, and growth of vascular tissue and new bone but also to reduce the compression modulus of solid metal as well to avoid the stress shielding effect. The compression modulus of human cortical bone is 89–164 MPa, while the elastic modulus of solid TC4 titanium alloy is up to 110 GPa. The selection of porous scaffolds significantly reduces the elastic modulus of materials. In this study, finite element analysis and biomechanical testing were carried out on the prepared 3D-printed titanium alloy porous scaffold. The compression moduli of the prepared 3D-printed titanium alloy porous scaffolds were 116.91 ± 0.01 and 174.29 ± 2.21 MPa, respectively, which was significantly lower than that of solid titanium alloy and close to the compression modulus of human cortex bone. Pobloth et al. demonstrated the necessity of creating mechanobiologically optimized Ti alloy scaffolds. A relatively soft scaffold led to regeneration in a large segmental bone defect in sheep, promoting endochondral and intramembranous bone formation [23]. Gao et al. performed a simulation study on mechanobiological optimization of a 3D titanium-mesh implant for mandibular large defects and reported that the optimized implant can provide an excellent mechanical environment for bone regeneration, achieving a long-term stability and occlusal reconstruction with defects [24].

In the in vitro biocompatibility experiment, the two groups of porous scaffolds with different unit structures showed no obvious cytotoxicity, good biocompatibility, and good cell morphology. There was no significant difference in the proliferation of cells on the scaffolds of the two groups. Wang et al. determined that an irregular pore size in scaffolds confers better osteogenesis and vascularization effects than a regular pore size in scaffolds [25]. Triangular, rectangular, and elliptic pores support angiogenesis and cause faster cell migration because the greater curvature helps to produce a larger bone volume compared with scaffolds with aligned patterns [26]. However, the surface of the scaffolds in group A was more conducive to cell adhesion than that in group B probably because the surface area of the underside of group B scaffolds was smaller, resulting in more cell adhesion inside the scaffolds or at the bottom of the orifice plate. In addition, the quantitative results of ALP staining showed that the ability of the scaffold in group A to promote bone differentiation was stronger than that in group B. Van Bael et al. found that the amount of pore occlusion was higher on scaffolds with hexagonal pores. When larger pores were used, cells were spread on the strut surface [27]. In other words, hexagonal pores facilitated cell growth because of higher number of corners and the short distance between the two arches in the corners, particularly in hexagonal pores [26]. Wu et al. reported that a more apparent anti-inflammatory microenvironment was generated by the hexagonal pore scaffold than the triangular one [28]. In addition, the accuracy of each SLM machine varies considerably, and the designed structures, especially at microscale, may be difficult to reproduce precisely.

The article "In Vitro and In Vivo Analysis of the Effects of 3D-Printed Porous Titanium Alloy Scaffold Structure on Osteogenic Activity" was published in 2022. Journal: Biomed Res Int.

In the in vivo experiment of rabbit femur defect repair, micro-CT three-dimensional images and quantitative results of new bone growth showed that although there was no significant statistical difference in new bone mass between the two groups, the data of group A were higher than that of group B. Fluorescence markers and VG staining results for hard tissue sections showed that the bone integration ability of new bone inside the scaffolds in group A was higher than that in group B, while VG staining results showed that the percentage of new bone area in the scaffolds in group A was higher than that in group B, indicating greater promotion of bone differentiation. These results indicate that the hollow hexagonal prism structure of the porous scaffold was better able to promote bone differentiation and bone integration than the triangular prism structure.

Based on the results of in vitro and in vivo studies, the porous scaffold shape had no obvious influence on cell activity and proliferation. The hexagonal prism unit structure had better ability to promote bone differentiation and bone integration than the triangular prism unit structure, possibly due to errors and spatial resolution. As a result, the surface shape of the hexagonal prism unit structure was closer to a circle, and the included angle between the beams was circular, which is more conducive to the attachment and spread of cells. Moreover, its larger surface area can increase the area of cell adhesion and make the cells accept more mechanical stimulation.

With continued development, the accuracy of the SLM technique is expected to be further improved; i.e., the geometries of created scaffolds will better match the designed geometries. Such deviation may not determine the effect of the geometry precisely, and the influence of other complicated geometries should be further explored.

## 5. Conclusions

Porous titanium alloy scaffolds with different unit structures were successfully prepared by SLM technology. The two scaffolds made of Ti6Al4V had compression moduli similar to that of human cortical bone. Cell adhesion was facilitated by hollow hexagonal prism than triangular prism structures. The number of cells adhered to both groups of scaffolds increased with culture time, and no significant difference in cell adhesion was found. Additionally, the osteogenic ability of the hollow hexagonal prism structure was stronger than that of triangular prism structure on the 12th day after culture. The in vivo tests showed that all scaffolds remained in good shape after implantation, and no obvious inflammatory reaction or infection in surrounding tissues was found. At week 12, the percentage of new bone area in the scaffold with the hollow hexagonal prism structure was higher than that in the scaffolds with the triangular prism structure. Thus, the hollow hexagonal prism structure of porous scaffolds can promote osteogenic differentiation and osseointegration better than the triangular prism structure. This work provides experimental results as well as insights into how two different structures influence the bone regeneration ability of titanium scaffolds.

The article "In Vitro and In Vivo Analysis of the Effects of 3D-Printed Porous Titanium Alloy Scaffold Structure on Osteogenic Activity" was published in 2022. Journal: Biomed Res Int.

## Figures and Tables

**Scheme 1:** Flow chart of the study.

**Figure 1:** (a, b) Three-dimensional digital model drawing of two kinds of porous structures with hollow hexagonal prism and hollow triangular prism element structure. (c) The finite element analysis software ANSYS simulates the stress of the support.

**Figure 2:** Images of 3D-printed porous titanium alloy scaffolds with two unit structures. Specifications: (a) bottom diameter 10 mm and thickness 5 mm (in vitro experiment) and (b) bottom diameter 5 mm and thickness 10 mm (in vivo experiment).

**Figure 3:** (a–c) Surface morphologies of 3D-printed porous titanium alloy scaffold. (d) Surface energy spectrum analysis (EDS) of 3D-printed porous titanium alloy scaffold. (e) X-ray diffraction (XRD) of 3D-printed porous titanium alloy scaffold.

**Figure 4:** Surface osteoblast adhesion results of 3D-printed titanium alloy porous scaffolds (multiple: ×200). (a) Group A. (b) Group B. (c) Quantitative analysis of surface osteoblast adhesion on 3D-printed porous titanium alloy scaffolds. ^∗^*P* < 0.05. (d, e) SEM image of surface osteoblast adhesion results of 3D-printed titanium alloy porous scaffolds. (f, g) Staining results of live and dead osteoblasts adhered to 3D printing porous titanium alloy scaffolds (multiple: ×200). (d, f) Group A. (e, g) Group B. (h) Proliferation results of cells adhered to scaffolds. (i) Quantitative results of ALP production by cells adhered to scaffolds. ^∗^*P* < 0.05.

**Figure 5:** (a) X-ray examination results of femur samples after scaffold implantation. (b) Micro-CT 3D reconstruction results. Yellow is bone tissue, and white is porous titanium alloy scaffold. (c) Results of new bone tissue parameters by micro-CT scanning in scaffold. (d) Fluorescent labeling results of newborn bone tissue in titanium alloy porous scaffold (multiple: ×200). Calcein labeled new bone tissue in green and titanium alloy material in black. (e) VG staining results of new born bone tissue in porous titanium alloy scaffold (multiple: ×200). Red is mature new bone tissue, brown gray is bone marrow tissue, and black is titanium alloy material. (f) Percentage of new bone area in porous titanium alloy scaffolds of the two groups. ^∗^*P* < 0.05 and ^∗∗^*P* < 0.01.

The article "In Vitro and In Vivo Analysis of the Effects of 3D-Printed Porous Titanium Alloy Scaffold Structure on Osteogenic Activity" was published in 2022. Journal: Biomed Res Int.

## Data Availability

The data that support the findings of this study are available from the corresponding authors upon reasonable request.
